The article "Internet of Things-Based Ultrasound-Guided Erector Spinae Plane Block Combined with Edaravone Anesthesia in Thoracoscopic Lobectomy" was published in 2021. Journal: J Healthc Eng.

# Internet of Things-Based Ultrasound-Guided Erector Spinae Plane Block Combined with Edaravone Anesthesia in Thoracoscopic Lobectomy

**DOI:** 10.1155/2021/9510783

**Published:** 2021-11-13

**Authors:** Xiuyan Wang, Xuan Zhou, Lin Li, Cuijie Liu

**Affiliations:** Department of Anesthesiology, Affiliated Hongqi Hospital of Mudanjiang Medical University, Mudanjiang 157011, Heilongjiang, China

## Abstract

This paper aimed to study the application value of Internet of Things (IoT) edge computing algorithm-based ultrasound-guided erector spinae plane block combined with edaravone anesthesia in thoracoscopic lobectomy. A total of 110 patients undergoing thoracoscopic resection were selected as subjects. The patients were anesthetized with erector spinae plane block combined with edaravone before surgery and underwent chest ultrasound scan. IoT edge computing algorithm was constructed and applied to ultrasound images of patients to enhance and denoise the images. It was found that, in different mixed noise mixtures (Gaussian noise 10% + speckle noise 90%; Gaussian noise 30% + speckle noise 70%), the edge computing algorithm can still maintain the edge information of the output image, showing better performance on edge information detection and denoising compared with the Prewitt and Canny operator. In addition, visual analog scale (VAS) scores decreased with postoperative time after edaravone anesthesia induction and erector spinae plane block lobectomy and reached the lowest level after five days. In short, erector spinae plane block combined with edaravone showed good sedative and analgesic effects on patients undergoing thoracoscopic lobectomy. Ultrasound images processed by IoT edge computing algorithm showed high accuracy in the identification of lung lesions, which was worth applying to clinical diagnosis.

## 1. Introduction

Lobectomy is mainly used for lobectomy of malignant tumors limited to the lung, pulmonary damage caused by tuberculosis, severe bullae, bronchiectasis, interstitial lesions, trauma, and dysplasia. Lobectomy is a kind of routine pulmonary resection [1]. The human body has five lobes in the chest cavity. The right lung is made up of the upper lobe, the middle lobe, and the lower lobe. The left lung is made up of two lobes, the upper lobe and the lower lobe. Lobectomy is suitable for lung cancer and irreversible lesions confined to the lung lobe. It mainly includes right upper lobectomy, right middle lobe lobectomy, right lower lobectomy, left upper lobectomy, and left lower lobectomy. If the lesion involves two lobes or the middle bronchus, upper-middle or lower-middle lobe, two-lobe lung resection is feasible [2]. In general, the quality of life of patients after surgery is good. In normal survival, postoperative patients need to pay attention to climate changes, keep warm, pay attention to diet, and avoid irritating gases [3]. In addition, patients need to exercise properly to enhance their resistance, closely observe their symptoms and signs, and go to the hospital for comprehensive examination and treatment as soon as possible if there is an abnormality [4, 5]. Thoracoscopic lobectomy means that, with the assistance of thoracoscopy, the surgeon only observes the situation in the thoracic cavity in real time through a TV screen and completes the operation through one to four hole-like incisions (without spreading the ribs) with the longest length not exceeding 5 cm. The veins, arteries, and bronchi are cut off anatomically to completely remove the lung lobes. At present, video-assisted thoracic surgery (VATS) lobectomy has basically matured and gained wide acceptance. The surgical technique is also gradually refined and perfected day by day [6, 7]. The National Comprehensive Cancer Network (NCCN) lung cancer treatment guidelines clearly point out that “VATS lobectomy is a viable option for resectable lung cancer,” which means that the role of thoracoscopic lobectomy for the treatment of benign lung lesions or early malignant lesions has been confirmed [8].

However, the postoperative pain of this type of surgery is relatively strong. Insufficient intraoperative anesthesia or insufficient postoperative analgesia will affect the patient's cough, sputum, and so on, which may easily lead to adverse events and affect the patient's recovery process. Edaravone is a new type of free radical scavenger, which can scavenge oxygen-free radicals, inhibit lipid peroxidation of cell membranes, and reduce tissue edema and damage. Studies have shown that edaravone can reduce the production of inflammatory factors in the human body and has a protective effect on the lungs of patients [9]. In recent years, an interfascial plane block technique has gradually been used clinically, that is, ultrasound-guided erector spinae plane block (ESPB). It was first applied to severe acute postoperative pain and neuropathic pain in 2016, and it was successful. Studies have shown that ESPB is easy to operate, has high safety, low error rate, good analgesic effect, and few adverse reactions, and shows broad clinical application prospects [10].

With the full integration and adoption of cutting-edge technologies such as big data, Internet+, AI, and Internet of Things (IoT), AI-assisted medicine has shown strong influence and vitality. It plays an important supporting role in deepening the reform of the medical and health system, accelerating the construction of “healthy China,” and promoting the development of the medical and health industry [11]. At present, medical imaging such as ultrasound (scanning the human body with ultrasound beam and obtaining images of internal organs by receiving and processing reflected signals) and magnetic resonance have gradually developed from auxiliary examination methods into the most important clinical diagnosis and differential diagnosis methods in modern medicine [12, 13]. Through big data plus artificial intelligence technology solutions, AI-assisted diagnosis and treatment adoptions are built, medical imaging data are modeled and analyzed, and conditions and lesions are analyzed to provide decision support for doctors and improve medical efficiency and quality [14, 15]. In this way, the high rate of misdiagnosis and missed diagnosis due to the limitation of doctors' experience in the field of medical imaging can be better solved, so did the long reading time, slow speed, and many other problems [16].

In the process of thoracoscopic lobectomy, some small pulmonary nodules cannot be accurately located during thoracoscopic surgery, and the boundary of pulmonary nodules is not easy to be identified. Ultrasonic guidance based on IoT edge detection algorithm was used to identify and locate hilar vessels and to surround small nodules in thoracoscopic lobotomy, to study the adoption value of the intelligent algorithm and ultrasound image in thoracoscopic lobectomy, aiming to provide more reference for the diagnosis and treatment of lobectomy and the sedation and analgesia methods of postoperative patients.

## 2. Materials and Methods

### 2.1. General Information

In this study, 110 patients who received thoracoscopic lobotomy in hospital from September 2019 to September 2020 were collected as subjects, including 58 male patients and 52 female patients aged 25∼68 years (43.7 ± 5.2 years on average). This study had been approved by the Medical Ethics Committee. The patients and their families understood the content and methods of the study and agreed to sign the corresponding informed consent.

Inclusion criteria were as follows: (i) patients who underwent lobectomy after prepathological and imaging diagnosis of lobectomy; (ii) patients aged between 45 and 65 years; (iii) patients with no pulmonary metastasis, mediastinal lymph node enlargement, or pleural hypertrophy; (iv) patients who had not received any other drugs or antibiotics recently; (v) patients with normal coagulation function and platelets.

Exclusion criteria were as follows: (i) patients with other system or organ lesions; (ii) patients who did not cooperate with treatment due to personal or other factors; (iii) patients with incomplete clinical data and medical history.

### 2.2. Patient Anesthesia and Surgical Methods

All patients were fasting and abstaining from drinking 6 h before anesthesia induction, and all vital signs were monitored before surgery, including heart rate, diastolic blood pressure, systolic blood pressure, pulse oxygen saturation, and mean arterial pressure. 0.5 mg/Kg edaravone was added to 100 mL normal saline, and the infusion was completed within 30 min. A conventional disinfection towel was taken from the surgical position, and an erector spinae plane block was performed under the guidance of ultrasound. The puncture was performed after local anesthesia with 1% lidocaine at the puncture site. Local anesthetic drugs were injected after a puncture to the designated location, and a two-point block was selected according to the intercostal incision. Each puncture site was injected with 10 mL of drugs, and 0.5 mg/Kg edaravone was used as an anesthetic. The results of nerve block were tested by alcohol cotton ball 10 minutes after injection.

In lobotomy, an incision was made in the fifth intercostal area between the midaxillary line and the anterior axillary line, approaching the hilum at a small angle to facilitate the operation of hand instruments along the longitudinal axis. During the operation, the hemodynamic indexes of patients were monitored in real time, and the corresponding vasoactive drugs were timely corrected in case of intraoperative hemodynamic instability.

All patients included in the study underwent lung ultrasound examination. The patient was placed in a lateral position, and a high-frequency linear array probe was used for sagittal scanning. After the T4 spinous process was positioned, the probe was moved 3–5 cm to the outside to show the T5 transverse process, pleura, and transverse costal ligament. The ultrasound images were interpreted by two attending physicians or imaging physicians with rich clinical experience. The specific location of pulmonary lesions, the maximum diameter of the lesion site, and hilar and mediastinal lymph node enlargement were mainly observed and analyzed by ultrasound.

### 2.3. IoT Edge Computing

The image edge generally refers to the position where the grayscale change rate of the image is the largest. Edge detection refers to the process of detecting edge points and edge segments from the image and describing the edge direction. The image is regarded as a binary function *f*(*x*, *y*), (*x*, *y*) is the position of the pixel, and *f*(*x*, *y*) is the gray value at that point so that the image is regarded as a curved surface. The edge of the image is the most drastically changing position on the curved surface, and this position is also the position of the local extreme point of the curved surface. The basic idea of the image segmentation method based on edge detection is determining the edge pixels in the image first. Then, these pixels are connected together to form the required area boundary.  Figure 1 shows the image edge type and its derivative curve law.

The brightness change of the image can be processed and enhanced by the difference between adjacent points. Differential processing of adjacent points in the horizontal direction can detect the brightness change in the vertical direction, that is, the horizontal edge detector (horizontal edge detector). Differential processing of adjacent points in the vertical direction can detect the brightness change in the horizontal direction, that is, the vertical edge detector (vertical edge detector). The expressions are shown in

(1) $$\begin{array}{c} E_{x}=\left|P_{x,y}-P_{x+1,y}\right|, \end{array}$$

(2) $$\begin{array}{c} E_{y}=\left|P_{x,y}-P_{x,y+1}\right|. \end{array}$$

Among them, *E*_*x*_ represents the vertical edge and *E*_*y*_ represents the horizontal edge. The horizontal edge detection operator and the vertical edge detection operator are combined, and the vertical edge and the horizontal edge can be detected at the same time, as shown in

(3) $$\begin{array}{c} E_{x,y}=\left|P_{x,y}-P_{x+1,y}+P_{x,y}-P_{x,y+1}\right|. \end{array}$$

From the above equation, equation (4) is obtained:

(4) $$\begin{array}{c} E_{x,y}=\left|2\times P_{x,y}-P_{x+1,y}-P_{x,y+1}\right|. \end{array}$$

If a pixel is inserted between two adjacent difference points to achieve this, it is equivalent to using two adjacent first-order differences as the new horizontal difference, as in

(5) $$\begin{array}{c} E_{xxx,y}=E_{xx+1,y}+E_{xx,y}=\left|P_{x+1,y}-P_{x,y}+P_{x,y}-P_{x-1,y}\right|=\left|P_{x+1,y}-P_{x-1,y}\right|. \end{array}$$

Here, *E*_*xx*_ represents the new level difference.

A gradient operator is defined by the method of first-order differentiation. The gradient is a vector, which indicates the direction of the most dramatic change in the gray level of the image.

(6) $$\begin{array}{c} \nabla f=\left(\frac{\partial f}{\partial x},\frac{\partial f}{\partial y}\right). \end{array}$$

The gradient can be expressed as

(7) $$\begin{array}{c} \left\|\nabla f\right\|=\sqrt{{\left(\frac{\partial f}{\partial x}\right)}^{2}+{\left(\frac{\partial f}{\partial y}\right)}^{2}}. \end{array}$$

The direction of the gradient is shown in

(8) $$\begin{array}{c} \theta =\left(\frac{\partial f/\partial y}{\partial f/\partial x}\right). \end{array}$$

In actual image processing, the difference method is used for calculation. However, the use of the differential method for edge detection must make the direction of the difference perpendicular to the direction of the edge. Therefore, it is necessary to perform difference calculations in different directions of the image, which increases the amount of calculation. Generally, the edges are divided into horizontal edges, vertical edges, and diagonal edges.

#### 2.3.1. Roberts Operator

The Roberts gradient operator uses the difference between the values of two adjacent pixels in the diagonal direction as a measurement standard, and its calculation method is shown in

(9) $$\begin{array}{c} G_{x}=f\left(i,j\right)-f\left(i-1,j-1\right), \end{array}$$

(10) $$\begin{array}{c} G_{y}=f\left(i-1,j\right)-f\left(i,j-1\right), \end{array}$$

(11) $$\begin{array}{c} \left|G\left(x,y\right)\right|=\sqrt{G_{x}^{2}+G_{y}^{2}}. \end{array}$$

Equation (11) is written in the form of convolution operation, and the convolution kernels are the following equations:

(12) $$\begin{array}{c} G_{x}=\left[\begin{array}{cc} -1 & 0\\ 0 & 1 \end{array}\right], \end{array}$$

(13) $$\begin{array}{c} G_{y}=\left[\begin{array}{cc} 0 & 11\\ 1 & 0 \end{array}\right]. \end{array}$$

#### 2.3.2. Prewitt Operator

The Prewitt operator combines the method of difference operation and neighborhood averaging, and its convolution template is shown in

(14) $$\begin{array}{c} G_{x}=\left[\begin{array}{ccc} -1 & 0 & 1\\ -1 & 0 & 1\\ -1 & 0 & 1 \end{array}\right], \end{array}$$

(15) $$\begin{array}{c} G_{y}=\left[\begin{array}{ccc} -1 & -1 & -1\\ 0 & 0 & 0\\ 1 & 1 & 1 \end{array}\right]. \end{array}$$

#### 2.3.3. Soble Operator

The two Soble operators are for detecting horizontal edges and detecting vertical edges. It weighs the influence of the position of the pixel, which can reduce the degree of edge blur. Since the Soble operator is a form of filter operator, it is used to extract the edge and can use the fast convolution function, which is simple and effective. However, the Soble operator does not strictly distinguish the main body of the image from the background; that is, it is not based on image grayscale processing.  Figure 2 shows the template of the Soble operator.

#### 2.3.4. Prewitt Edge Detection Operator

If the weights of the center pixels of the two Prewitt template operators are doubled, the well-known Soble edge detection operator is obtained. It is composed of two masks that determine the edge in a vector manner. Soble has better performance than other edge detection operators in the same period as the Prewitt operator (Figure 3).

### 2.4. Evaluation of Edge Detection Effect of Ultrasonic Images

Ultrasound uses the difference between echo and original sound waves to produce images. The ultrasonic wave will change after being reflected by the object. The change is related to the shape characteristics of the object, and the shape of the object is determined according to the reflected wave. Ultrasound is injected into the body through the organs and tissues with different acoustic impedance and different attenuation characteristics from the surface to the deep, resulting in different reflections and attenuations. However, the existing ultrasound imaging technology is susceptible to interference from image noise, and the detection effect of blur and discontinuous edges is not good. Therefore, the IoT edge detection algorithm processes the ultrasound image and then judges its blur and discontinuous edge detection effect on the ultrasound image by setting the direction of the edge detection and the edge gray threshold.

### 2.5. VAS Evaluation Criteria

VAS is used for pain assessment and is widely used in clinical practice. The basic method is to use a moving ruler about 10 cm long with 10 scales on one side, and the two ends are “0” and “10” points, respectively. 0 points mean no pain, and 10 points mean the most severe pain that is unbearable [17].

### 2.6. Statistical Methods

The data processing in this study was analyzed by SPSS 19.0 version statistical software, some measurement data were expressed by the mean ± standard deviation ($\bar{x}$ ± *s*), and the count data were expressed by the percentage (%). Pairwise comparison used analysis of variance. *P* < 0.05 indicated that the difference was significant.

## 3. Results

### 3.1. Lung Ultrasound Signs

Figure 4 shows the ultrasound signs of the lungs. In a normal lung ultrasound image, a hyperechoic line that slid back and forth with breathing motion was seen on the deep surface of the rib line, which was called the “pleural line.” When the ultrasound was projected perpendicularly to the pleura-lung surface, reverberation artifacts may appear, which were manifested as multiple echoes arranged at equal distances. Its intensity decreased successively, called “A line,” so the normal lung ultrasound image features were “slip sign” and “A line.”

### 3.2. Signal-to-Noise Ratio of the Output Image

The signal-to-noise ratio of the filtered image can represent the denoising effect of the algorithm on the image with noise. Figures 5 and 6 show the signal-to-noise ratio (SNR) of the output image processed by different filters under Gaussian noise 10% and speckle noise 90% and Gaussian noise 30% and speckle noise 70% of the noise mixed conditions, respectively. Under different mixed noise conditions and signal-to-noise ratio conditions, the edge detection algorithm can still better maintain the edge information of the output image, and the image enhancement effect was ideal.

### 3.3. Lung Ultrasound Edge Detection

Figure 7 shows the ultrasound images of the lung and the image after image enhancement and noise processing were performed by the edge detection algorithms of the Canny operator, Prewitt operator, and Soble operator. The improved filter of the edge detection algorithm can not only maintain the original texture details and edge information of the input and output images in the image processing process but also process and suppress the noise pollution of the background of the image and the internal noise of the organization to a higher degree. Moreover, the Soble operator had better edge detection performance than the Prewitt operator and Canny operator in the same period and had better edge information detection and denoising performance for ultrasound images.

### 3.4. Detection Rate of Lung Nodules by Three Edge Detection Operators

Figure 8 shows the comparison results of the detection rates of lung nodules of different sizes after the Canny operator, Prewitt operator, and Soble operator edge detection algorithms processed lung ultrasound images. For lung nodules smaller than 6 mm, the detection rates of the three edge detection operators were 90.98%, 87.53%, and 92.35%, respectively. For lung nodules from 6 to 30 mm, the detection rates of the three edge detection operators were 88.32%, 90.87%, and 95.44%, respectively. The detection rate of the Soble operator for lung nodules of different sizes was significantly higher than that of the Canny operator and Prewitt operator edge detection algorithm (*P* < 0.05).

### 3.5. VAS Score after the Patient's Operation

Figure 9 shows the visual analog score (VAS) of patients in different periods after thoracoscopic lobectomy.  Figure 9(a) shows the VAS score result in the resting state, and Figure 9(b) shows the VAS score result in the patient's exercise state. After edaravone was used for induction of anesthesia and lobectomy after erector spinae plane block, the patient's VAS score decreased with the prolongation of postoperative time. After five days, the patient's VAS score was reduced to a lower level.

## 4. Discussion

Edge detection of medical image is an important basis for image segmentation, object recognition, region shape extraction, and other image processing fields. In the process of image understanding and analysis, the first step is often edge detection to identify the points with obvious brightness changes in digital images [18]. The so-called edge refers to the set of pixels with sharp changes in the gray level of the surrounding pixels, which is the basic feature of the image. Edge exists between target, background, and region, which is the most important basis for image segmentation. As an indicator of position, edge is insensitive to changes in gray level, so it is an important feature of image matching [19]. Image edge contains the useful information used for identification in the image, which greatly reduces the amount of data, eliminates the irrelevant information, and retains the important structural attributes of the image. The use of edge detection technology for visual detection has become the latest trend in image sensor adoptions. In addition, as edge detection plays an important role in image analysis such as computer vision and ultrasound, it provides valuable feature parameters for people to describe or identify objects and to interpret images. Cao et al. [20] found that ultrasound-guided erector spinae plane block technology had the advantages of simple operation and high safety factor. In addition, ultrasound-guided erector spinae plane block lobectomy was performed with high recognition of intermuscular images and no risk of spinal cord injury compared with other blocking methods. Erector spinae plane block has a long duration of action and a wide range of action. To a certain extent, it can effectively shorten the hospital stay of patients undergoing lobectomy and accelerate the postoperative recovery speed, which has a high adoption value.

In this study, patients undergoing laparoscopic lobectomy were selected as subjects, and lung ultrasound examination was performed on the included patients. The ultrasonic image was filtered, enhanced, and denoised by IoT edge detection algorithm. Ultrasound images were processed and used in erector spinae plane block combined with edaravone anesthesia-induced lobectomy. It was found that, under different mixed noise conditions and SNR conditions, the edge detection algorithm can still maintain the edge information of the output image well and the image enhancement effect was good. The Soble operator had better edge detection performance than the Prewitt operator and Canny operator at the same period and had better edge information detection performance for ultrasonic images. Edge detection and filtering had a good effect on noise removal of ultrasonic images. The detection rate of the Soble operator for pulmonary nodules of different sizes was significantly higher than that of the Canny operator and Prewitt operator (*P* < 0.05). VAS scores decreased with postoperative time after edaravone anesthesia induction and erector spinae plane block lobectomy. After five days, the VAS score of the patients was reduced to a low level. The results of this study were in line with expectations. A number of previous studies have shown that erector spinal muscle plane block combined with edaravone has a positive sedative and analgesic effect on patients undergoing thoracoscopic lobectomy. Ultrasound images based on IoT edge computing algorithm are more accurate in the identification of lung lesions. This was similar to the results of Williams et al. [21], indicating that erector spinae plane block combined with edaravone anesthesia induction had good sedative and analgesic effects on patients undergoing thoracoscopic lobectomy, which also improved the prognosis of patients.

## 5. Conclusion

In this study, three edge detection algorithm models were constructed and applied in the ultrasound images of 110 patients with lung disease. The results found that the erector spinal muscle plane block combined with edaravone had a better sedative and analgesic effect on patients undergoing thoracoscopic lobectomy. The ultrasound image based on the IoT edge computing algorithm showed higher accuracy in identifying lung lesions, and it was worth applying to clinical diagnosis. The disadvantage was that it lacked comparison with other intelligent algorithms, and the representativeness was low. Therefore, in subsequent experiments, an improvement and optimization would be made in this area, and more in-depth exploration of this direction would be carried out. In summary, this study provided a reference for the application of intelligent algorithms such as edge detection in medical imaging.

## Figures and Tables

**Figure 1:** Image edge type and its derivative curve law. (a) Gray cross section-step shape; (b) gray cross section-thin line shape; (c) gray cross section slope gradient; (d) first-order differential-step shape; (e) first-order differential-thin line shape; (f) first-order differential-slope gradient shape; (g) second-order differential-step shape; (h) second-order differential-thin line shape; (i) second-order differential-slope gradient shape.

**Figure 2:** The template of the Soble operator. (a)*G*_*x*_; (b)*G*_*y*_.

**Figure 3:** Template of Prewitt operator. (a) The Prewitt operator template Mx; (b) the Prewitt operator template My.

**Figure 4:** Ultrasound signs of the lungs. (a) A line; (b) B line; (c) normal; (d) mild-to-moderate interstitial edema; (e) severe interstitial edema and alveolar edema; (f) lung consolidation.

**Figure 5:** Signal-to-noise ratio of the output image of the edge detection filter (Gaussian noise 10%; speckle noise 90%).

**Figure 6:** Signal-to-noise ratio of the output image of the edge detection filter (Gaussian noise 30%; speckle noise 70%).

**Figure 7:** Ultrasonic edge detection of lungs. (a) The original image; (b) the image contaminated by noise; (c–e) edge detection and image processing of Canny operator, Prewitt operator, and Soble operator, respectively.

**Figure 8:** Detection rate of lung nodules by three edge detection operators. Note: ^*∗*^ means significant difference compared to Canny operator (*P* < 0.05); # means significant difference compared to Prewitt operator (*P* < 0.05).

**Figure 9:** Postoperative VAS score of patients. (a) The VAS score in the resting state; (b) the VAS score in the exercise state.

## Data Availability

The data used to support the findings of this study are available from the corresponding author upon request.
